The article "Observation on the Effect of Bone Grafting Alone and Guided Tissue Regeneration Combined with Bone Grafting to Repair Periodontal Intraosseous Defects" was retracted in 2023. Reasons: unreliable results or conclusions; concerns about the data; concerns about the peer review; concerns about the citations.

# Observation on the Effect of Bone Grafting Alone and Guided Tissue Regeneration Combined with Bone Grafting to Repair Periodontal Intraosseous Defects

**DOI:** 10.1155/2021/1743677

**Published:** 2021-10-12

**Authors:** Yongping Yuan, Jiajia Zhao, Nv He

**Affiliations:** ^1^Oral Teaching and Research Office, Ningbo Colloge of Health Sciences, Ningbo, Zhejiang 315100, China; ^2^Department of Dental, Zhuji People's Hospital, Zhuji, Zhejiang 311800, China

## Abstract

**Objective:**

To investigate the curative effect of guided tissue regeneration (GTR) combined with bone grafting and improve the aesthetic appearance of patients' gingiva.

**Methods:**

A total of 86 patients with periodontal intraosseous defects were selected from February 2019 to February 2021. All the patients were divided into a control group and an observation group according to the random number table, with 43 patients in each group. Bone grafting was performed in the control group, while GTR was additionally used in the observation group on the basis of the control group. The surgical data and follow-up data were collected and organized. The alveolar bone mineral density, the change in the height of the bone defect, plaque index (PLI), sulcus hemorrhage index (SBI), PD, gingival recession (GR), clinical attachment loss (CAL), and other relevant data of the two groups in 6 months before and after surgery were compared. Six months after surgery, the cosmetic morphology of the patient's gums in the soft tissues around her teeth was evaluated.

**Results:**

Six months after surgery, the alveolar bone density of patients in two groups increased compared with that before surgery, and the height of the bone defect decreased compared with that before surgery. The alveolar bone density of the observation group was higher than that of the control group, and the height of the bone defect was lower than that of the control group (*P* < 0.05). Six months after surgery, the PLI, SBI, PD, and CAL of patients in both groups were lower than those before surgery, while the GR was higher than that before surgery. PD and CAL values in the observation group were lower than those in the control group, and GR was higher than that in the control group (*P* < 0.05). Six months after surgery, there was no significant difference in PLI and SBI scores between the two groups (*P* < 0.05). Six months after surgery, the gingival cosmetic scores of the two groups of patients were higher than those before surgery. The observation group was higher than the control group (*P* < 0.05).

**Conclusion:**

GTR combined with bone grafting has a good effect in the repair of periodontal intraosseous defects and can effectively promote the reconstruction and recovery of periodontal intraosseous defects in patients. At the same time, it can significantly improve the aesthetic appearance of patients' gums, with good clinical application value.

## 1. Introduction

Periodontal disease is a common disease in oral surgery, especially in the periodontal supporting tissues (gums, periodontal ligament, alveolar bone, and cementum). The incidence rate is high, manifested as gingival swelling and bleeding, which affects the quality of life of patients, which is one of the main causes of adult dentition defects [1, 2]. The periodontal intraosseous defect is a serious clinical symptom caused by periodontal diseases, such as gingival disease and periodontitis. If not treated in time, it can lead to alveolar bone resorption and defect, periodontal attachment loss, and teeth loosening and falling off [3, 4]. Periodontal bone defects affect the masticatory function and aesthetic appearance of patients and increase their physiological and psychological pressure. Therefore, the treatment of periodontal disease should focus on eliminating the source of infection and local stimulation factors and pay attention to the repair of periodontal tissue defects and the recovery of normal morphology and function. Bone grafting is to repair periodontal defects by transplanting materials (bone or bone substitutes), so as to restore the anatomical morphology of the alveolar bone and the function of periodontal tissue [5, 6]. The complete concept of periodontal attachment is to establish a complete periodontal tissue, including the cementum, periodontal ligaments, alveolar bone, and connective tissue attachment. At present, one of the hot spots in the treatment of periodontal intraosseous defects is the treatment that can effectively promote periodontal tissue regeneration and increase periodontal attachment. Bone grafting is a method to promote new bone formation and repair the alveolar bone defects caused by periodontitis by using bone or bone substitutes. Guided tissue regeneration (GTR) was put forward by Melcher in 1976, and it was used in periodontal surgery. Collagen membrane acts as a physical barrier, which separates different tissues by surgery. Then, depending on the mechanical barrier of the membrane, GTR can selectively guide the periodontal regenerated cells to grow back to the damaged area, so as to realize the attachment and proliferation of the damaged periodontal area [7, 8]. At present, clinically, when the thickness of the buccal bone plate in the alveolar socket is less than 1.5–2.0 mm (mostly located in the anterior aesthetic area) and, at the same time, there is more than one bone wall defect or missing in the alveolar socket, GTR may be considered for patients with few teeth reserved and patients with bone reserved for future restoration. A large number of studies in the literature have confirmed that GTR is a mature and stable method for vertical bone increment [9, 10]. In this study, GTR combined with bone grafting was used to treat patients with the periodontal intraosseous defect and compared with patients with bone grafting alone to explore the effect of GTR combined with bone grafting on periodontal intraosseous defects and to provide reference for clinical practice.

## 2. Materials and Methods

### 2.1. General Materials

A total of 86 patients with periodontal intraosseous defects admitted to our hospital from February 2019 to February 2021 were selected. The inclusion criteria were as follows: (1) the basic periodontal treatment has been completed for 4 weeks. The lesions mainly involve a single tooth surface of the anterior or posterior teeth, and the periodontal probing depth (PD) is not less than 6 mm; (2) the panoramic film shows that the alveolar bone has vertical absorption; (3) the angle of the bone defect is less than 60°, and the vertical depth of the bone pocket is greater than 3 mm; (4) there is no contraindication to periodontal surgery, and the patient has informed consent. The exclusion criteria were as follows: (1) combined diabetes or osteoporosis; (2) combined with severe immunodeficiency or coagulation dysfunction; (3) accompanied by habitual bruxism. All patients were divided into the control group and observation group by the random number table method, each with 43 patients. There was no statistically significant difference between the two groups of general information (*P* < 0.05), and they were comparable, as shown in Table 1.

### 2.2. Research Method

Bone grafting was performed in the control group. First, the skin flap was transferred through a modified periodontal incision, and curettage was completed after the diseased tissue was exposed. The root surface was trimmed and treated to make it smooth, rinsed, and washed with normal saline, and bone meal was then implanted into the bone defect area at a height up to the level of the bone pocket, and appropriate pressure was applied to help it compress and shape, thereby restoring the shape of the periodontal bone as much as possible. The gingival flap was sutured with an absorbable suture, and suppository was used for external application. The observation group was treated with GTR combined with bone grafting. The femoral bone meal was implanted into the defect at a height up to the level of the bone pocket and appropriately compressed to restore the periodontal bone morphology as far as possible. The collagen membrane was trimmed to an appropriate size according to the periodontal bone morphology, and the bone defect was covered with the collagen membrane to ensure that the collagen membrane covered the normal alveolar bone of about 2.5 mm. After the complete coverage and anastomosis of the bone defects were ensured, the collagen membrane was applied to the root surface and crown to avoid overlapping or folding and then sutured and fixed to the affected tooth. Finally, the absorbable suture was used to firmly restore and suture the gingival flap. When restoring the gingival flap, the operation area was completely covered, and the gingival flap was tightly sutured without exposing the membrane. After compression hemostasis, periodontal plug treatment agent was used to protect the wound.

The surgical data and follow-up data of the patients were collected and sorted, and then the relevant data of the two groups before and 6 months after surgery were compared, such as alveolar bone density, changes in bone defect height, plaque index (PLI), sulcus bleeding index (SBI), PD, gum recession (GR), and clinical attachment loss (CAL). At 6 months after surgery, the soft tissue around the patient's teeth was evaluated for gingival cosmetic morphology. The higher the score, the better the aesthetic effect. The scoring criteria are shown in Table 2.

## 3. Statistical Method

SPSS 22.0 software is used for data processing, the experimental data are expressed in mean ± standard deviation, and the count data are expressed in rate. The pairwise comparison of measurement data between groups is analyzed by the *t*-test, and count data are analyzed by *χ*^2^ test. The test level is *α* = 0.05, and *P* < 0.05 indicates that the difference is statistically significant.

## 4. Results

### 4.1. Results of Surgery and Follow-Up Examinations in the Two Groups

On the postoperative day, the teeth of all patients achieved good initial stability. Reexamination at 6 months after surgery showed that the defect of 86 patients was not loosened or shedding, osseointegration was good, mucosa was healthy, and there was no pain or paresthesia in the defect. During the period, there was no infection, bone meal discharge, etc. Clinical follow-up examinations of patients in typical cases from the day of surgery to 12 months after surgery showed that the bone bonds at the defects were good, the mucosa was healthy, and there was no loosening or dropping out. All the implants functioned well. The results of the imaging examination showed that the osseointegration of the defect was good, and there was no transmission shadow around it, as shown in Figure 1.

### 4.2. Comparison of Alveolar Bone Density and Bone Defect Height between the Two Groups

At 6 months after surgery, the alveolar bone density of the two groups of patients was higher than that preoperative, and the height of the bone defect was lower than that preoperative. The alveolar bone density of the observation group was higher than that of the control group, and the height of the bone defect was lower than that of the control group; the differences were statistically significant (*P* < 0.05), as shown in Figure 2.

### 4.3. Comparison of PLI, SBI, PD, GR, and CAL between the Two Groups

At 6 months after surgery, the PLI, SBI, PD, and CAL of the two groups of patients were lower than those preoperative, and the GR was higher than that preoperative. The PD and CAL of the observation group were lower than those of the control group, and the GR was higher than that of the control group. The differences were statistically significant (*P* < 0.05). At 6 months after surgery, there was no significant difference in PLI and SBI between the two groups of patients (*P* > 0.05), as shown in Figure 3.

### 4.4. Comparison of Gingival Cosmetic Morphology Scores between the Two Groups

At 6 months after surgery, the scores of gingival cosmetic appearance of the two groups of patients were higher than preoperative. The observation group was higher than the control group, and the difference was statistically significant (*P* < 0.05), as shown in Figure 4.

## 5. Discussion

In recent years, with the rapid development of medical technology, more and more scholars are concerned about the importance of periodontal ligament. Gingival disease and chronic periodontitis are both periodontal diseases with a high incidence, which can be manifested as gingival swelling and bleeding, and are also one of the important reasons for the periodontal intraosseous defect [11]. The development of chronic periodontitis will cause the reduction or loss of chewing function to a certain extent, and it is the “number one killer” of oral health. At present, the prevalence of periodontal disease in China is high, which has seriously affected the quality of life. For patients with moderate to severe chronic periodontitis with periodontal bone defects, basic periodontal treatment cannot always achieve the desired results [12, 13]. Clinically, periodontal intraosseous defects are often treated by surgery. Among them, bone grafting is a method for treating inflammation and destruction of the periodontal soft tissue and periodontal bone, and its curative effect is exact [14]. With the development of stomatology and the research and development of new materials, how to promote the regeneration of periodontal tissue, restore the function of periodontal tissue, give attention to gingival aesthetics, and eliminate the symptoms of infection and destruction on the basis of simple bone grafting has become a new direction for the clinical treatment of the periodontal intraosseous defect [15, 16].

GTR separates the gingival connective tissue epithelium from the exposed root surface through a physical barrier film such as the collagen membrane, which delays the root migration of the epithelium and promotes the reattachment and growth of cells from the periodontal membrane. Combined with bone transplantation, the bone substitutes were implanted into bone defects to promote blood vessel regeneration and guide attachment of periodontal precursor cells [17, 18]. In this study, all patients had good initial stability of their missing teeth the next day after surgery. Follow-up observation showed that all patients had no defect loosening or falling off, good osseointegration, healthy mucous membrane, and no pain or abnormal sensation at the defect. The results of imaging examination showed that the osseointegration of the defect was good, and there was no transmission shadow around it. It showed that bone grafting alone and GTR combined with bone grafting achieved good results in patients with the periodontal intraosseous defects, and there was no obvious adverse reaction. The results of this study also showed that 6 months after surgery, the alveolar bone density and the height of bone defects in the two groups were better than those before the operation, and the observation group was significantly better than the control group. The collagen membrane used in GTR is soft, is easy to shape, and has good histocompatibility. Moreover, it is an absorbable film, which can be degraded and absorbed by itself and does not need to be operated again. At the same time due to its material characteristics, weak mechanical strength is prone to collapse, which affects the space of the osteogenic area and leads to insufficient bone formation [19]. Some complications mentioned in the study are the early degradation of the absorbable membrane, which will reduce its barrier function, lead to the gingival flap to moving to the crown after the operation, and lead to the loss of keratinized gingival width and thickness [20]. Therefore, GTR is often combined with bone grafting; that is, bone or bone replacement material is implanted into the periodontal bone defect, and the implanted bone acts as a scaffold for degradation and absorption, and finally, the autologous bone grows in to restore the structure and function of the periodontal supporting tissue. The GTR combined with bone grafting can support the collagen membrane to achieve isolation and provide enough space for periodontal bone regeneration. On the one hand, the regenerated bone tissue can grow into the concave part of the bone with the periodontal defect and come into direct contact with the root surface. On the other hand, it can increase the regeneration ability of the bone tissue and promote the repair effect [21].

The results of this study showed that, at 6 months after surgery, PLI, SBI, PD, CAL, and GR in the two groups were better than those before surgery. PD, CAL, and GR in the observation group were significantly better than those in the control group. Bone powder is a carbonate apatite crystal that can be used to fill the defective alveolar bone, but it is difficult to model, and it is often necessary to use a buccal-lingual mucoperiosteal valve or a wandering gingival valve to close the extraction wound, which will increase the trauma and reduce the keratotic gingiva. GTR combined with bone grafting not only played an important role in the reconstruction and recovery of bone defect tissue but also significantly promoted the healing of soft tissues. A certain thickness of highly mature gingival soft tissue around the bone defect plays a positive role in alleviating inflammation and promoting bone integration [22, 23]. After the operation, our doctors discussed the details of the operation repeatedly and summarized the experience of the operation. They concluded that treating the root surface with tetracycline aqueous solution could effectively remove the smear layer and antibacterial effect and, at the same time, improve the biocompatibility of the root surface and promote the formation of new attachments. This was an important part of the surgical process.

With people's pursuit of oral health and beauty, the cosmetic shape of gums has gradually gained attention in the restoration of the periodontal intraosseous defects [24]. In this study, the gingival cosmetic appearance score of the observation group was significantly higher than that of the control group at 6 months after surgery. It showed that the GTR combined with bone grafting was better than bone grafting alone in improving the aesthetics of the patients' gums, which might be related to its promotion of soft tissue healing and the good integration of soft tissues [25]. Hydroxyapatite is a kind of bone substitute material for bone transplantation, which can enhance the proliferation and adhesion activity of gingival fibroblasts. In addition, hydroxyapatite has the role of a scaffold, which can protect the collagen membrane from displacement or deformation caused by the compression of foreign tissues.

In conclusion, the GTR combined with bone grafting has a good effect in repairing periodontal intraosseous defects and can effectively promote the reconstruction and recovery of the periodontal intraosseous defects in patients. At the same time, it can significantly improve the gingival aesthetics of patients, which has good clinical application value.

## Figures and Tables

**Figure 1:** Imaging results of the control group patients during follow-up. (a) Oral picture before operation. (b) Oral picture 6 months after surgery. (c) Oral picture 12 months after surgery. (d) Image picture after surgery. (e) Image picture 6 months after surgery. (f) Image picture 12 months after surgery.

**Figure 2:** Alveolar bone density and bone defect height between the two groups. *Note.* Compared with the same group preoperative, ^*∗*^*P* < 0.05; compared with the control group, ^#^*P* < 0.05.

**Figure 3:** PLI, SBI, PD, GR, and CAL between the two groups. *Note.* Compared with the same group preoperative, ^*∗*^*P* < 0.05; compared with the control group, ^#^*P* < 0.05.

**Figure 4:** Gingival cosmetic morphology scores between the two groups. *Note.* Compared with the same group preoperative, ^*∗*^*P* < 0.05; compared with the control group, ^#^*P* < 0.05.

**Table 1:** Comparison of general information of the two groups (*n*, $\bar{x}$ ± *s*).

Group	Male/female	Age (years)	Number of bone defects			Location		
			1	2	3	Left	Right	Bilateral
Control group (*n* = 43)	20/23	41.52 ± 6.84	31	9	3	15	13	15
Observation group (*n* = 43)	19/24	42.13 ± 5.61	29	12	2	13	14	16
*t*/*χ*^2^ value	0.047	0.452		0.695			0.212	
*P* value	0.829	0.652		0.706			0.899	

**Table 2:** The scoring standard of the cosmetic gingival morphology.

Project	0 points	1 point	2 points
Proximal, middle, and distal gingival papillae	Lack	Incomplete	Complete
Soft tissue level	<1 mm	1-2 mm	>2 mm
Soft tissue color	Significant differences	Severe difference	No differences
Soft tissue texture	Significant differences	Severe difference	No differences
Soft tissue contour	Discord	Relative harmony	Natural harmony
Alveolar bone defect	Obvious defect	Mild defect	No defect

## Data Availability

The data used during the current study are available from the corresponding author upon request.
